RETRACTED

# MicroRNA-223 decreases cell proliferation, migration, invasion, and enhances cell apoptosis in childhood acute lymphoblastic leukemia via targeting Forkhead box O 1

**DOI:** 10.1042/BSR20200485

**Published:** 2020-10-06

**Authors:** Chunyu Li, Tana Zhao, Lei Nie, Yanhong Zou, Quan Zhang

**Affiliations:** 1 Department of Pediatrics, The First Affiliated Hospital of Jiamusi University, No. 348 dexiang Street, Jiamusi City, Heilongjiang Province 154002, China; 2 Department of Gastroenterology, Jiamusi Central Hospital, No. 256, Zhongshan Street, Xiangyang District, Jiamusi City, Heilongjiang Province 154002, China

**Keywords:** acute lymphoblastic leukemia, cell apoptosis, cell proliferation, FOXO1, migration and invasion, miR-223

## Abstract

**Objective:** Acute lymphoblastic leukemia (ALL) is a frequent malignancy in childhood. The present study was aimed to investigate the effect of miR-223 in ALL and its underlying molecular mechanisms.

**Methods:** The mRNA expression of miR-223 and FOXO1 was detected by qRT-RCR in ALL children. The correlation between miR-223 and clinical indexes of ALL was determined. CCRF-CEM and NALM-6 cells were transfected with miR-223 mimic and miR-223 inhibitor, respectively. The proliferation, apoptosis, invasion and migration of CCRF-CEM and NALM-6 cells were measured by MTT, flow cytometry and transwell assay. The protein expression of FOXO1 was detected by Western blot. Additionally, dual-luciferase reporter and RNA pull-down assay were performed to investigate the target gene of miR-223 and validate their targeting relationship.

**Results:** The mRNA expression of miR-223 was markedly down-regulated in ALL, but FOXO1 was up-regulated. The protein expression of FOXO1 was highly expressed in CCRF-CEM and NALM-6 cells. The expression of miR-223 was related to WBC, PLT, RBC and risk stratification. Overexpression of miR-223 not only inhibited cell proliferation, migration and invasion, but also induced cell apoptosis. Importantly, FOXO1 was a target gene of miR-223 in ALL cells. Silencing of FOXO1 reversed the effects of miR-223 inhibitor on cell proliferation, migration, invasion and apoptosis in ALL.

**Conclusions:** miR-223 could inhibit cell proliferation, migration and invasion, and promote apoptosis by targeting FOXO1 in ALL.

## Introduction

Acute lymphoblastic leukemia (ALL) is a frequent malignancy in childhood, accounting for 75–80% of children with acute leukemia [1]. The ALL is characterized by infiltration of the bone marrow and accumulation of lymphoblasts in liver, spleen and lymph nodes [2]. Most all patients can achieve long-term disease-free survival through standardized treatment, while there are still some ALL children with recurrence are difficult to achieve remission [3]. Most of survivors of ALL children exhibit poor prognosis after their initial diagnosis, and early countermeasures to decrease late therapy-related effects is the main challenge in the treatment of ALL children [4]. Therefore, it is urgent to explore new strategies for the treatment of ALL children.

RETRACTED

Dysregulation of microRNAs (miRNAs) are closely related to the tumorigenesis in several human cancer types including ALL [5]. MiRNAs play a key role in inhibiting ALL and chronic lymphocytic leukemia (CLL), and have a good application prospect in targeted molecular therapy and prognosis evaluation [6]. Accumulating evidence has confirmed that miRNAs have important effects on biological processes of lymphocytic leukemia, including cell proliferation, apoptosis, cycle and carcinogenesis [7,8]. Importantly, miR-223 plays an important role in lymphocytic leukemia. For example, up-regulation of miR-223 can attenuate the proliferation and colony formation of ALL cells [9]. The miR-223 expression was down-regulated at new diagnosis and up-regulated at complete remission in ALL children [10]. Silencing of miR-223 is related to poor prognostic factors and disease aggressiveness in CLL [11]. However, the underlying mechanism of miR-223 in the progression of ALL children remains limited.

Forkhead box class O (FOXO) is a subfamily of transcription factors that acts as a target involved in cell differentiation and apoptosis [12]. FOXO1 can be regulated by miRNAs since the 3′ UTR contains miRNA-binding sites [13,14]. Previous research has been demonstrated that FOXO1 is introduced as a therapeutic target for patients with ALL [15,16]. Importantly, FOXO1 expression and cell proliferation have been proved to be regulated by miR-223 in colorectal cancer cells and hepatoma cells [17]. However, the specific regulatory relationship between miR-223 and FOXO1 remains undefined in ALL children.

In the present study, we examined the effects of miR-223 on proliferation, migration, invasion and apoptosis of ALL cells. We also verified the targeting relationship between miR-223 and FOXO1. Our research may discover a hopeful therapeutic target for ALL children, and reveal the underlying mechanisms for ALL treatment.

## Materials and methods

### Patients and tissue samples

From January 2016 to December 2018, total bone marrows from 59 ALL children were collected in our hospital. The ALL in the present study were diagnosed by ‘National recommendations for diagnosis and treatment of children with ALL (fifth revised draft)’. ALL children included 17 children with standard risk (SR), 25 children with intermediate risk (IR) and 17 children with high risk (HR). Meanwhile, 30 children without malignant hematologic diseases in our hospital were collected as controls case (Control). The present study was approved by the Ethics Committee belonging to our hospital. In addition, all patients involved provided informed consent.

RETRACTED

### Cell cultures

Human ALL cells line, CCRF-CEM and NALM-6 cells were supplied by American Type Culture Collection. CCRF-CEM cells and NALM-6 cells were cultured in Dulbecco’s Modified Eagle Medium complemented with 10% fetal bovine serum (FBS) and 1% streptomycin/penicillin in a 5% CO_2_ incubator at 37°C.

### Quantitative real-time polymerase chain reaction (qRT-PCR)

Total RNA from human ALL cells line was extracted by TRIZOL (Invitrogen, Carlsbad, CA, U.S.A.) and was reverse-transcribed into cDNA by Takara PrimeScript RT Reagent Kit (Takara, Otsu, Japan). PCR reaction was performed on ABI 7500HT Fast Real-Time PCR System (Applied Biosystems, Waltham, MA, U.S.A.) with the following conditions: 95°C for 3 min, 40 cycles of 95°C for 15 s and 60°C for 30 s. Relative expression was calculated by the 2^−ΔΔCt^ method. Primers used in the present study were listed in Table 1. β-Actin and U6 were respectively used as internal controls of FOXO1 and miR-223.

**Table 1:** Primers sequences

Primers	Sequences
miR-223	Forward: 5′-CAGCACCACTGAATCACAGA-3′
	Reverse: 5′-GTGCAGGGTCCGAGGT-3′
U6	Forward: 5′-CTCGCTTCGGCAGCACA-3′
	Reverse: 5′-AACGCTTCACGAATTTGCGT-3′
FOXO1	Forward: 5′-AAGGACCCAGCCCTCAAGAA-3′
	Reverse: 5′-TGCTCTAGAGCAATACAGCAAGTTACC-3′
si-FOXO1	Forward: 5′-CAGCACCACTGAATCACAGA-3′
	Reverse: 5′-AGTATGAAACATCCCCACAGGG-3′
β-Actin	Forward: 5′-ACACCTTCTACAATGAGCTG-3′
	Reverse: 5′-CTGCTTGCTGATCCACATCT-3′

### Cell transfection

The miR-223 mimic, negative control (NC)-mimic, miR-223 inhibitor and NC-inhibitor were bought from GenePharma (Shanghai, China). FOXO1 siRNA-1 (si-FOXO1-1), si-FOXO1-1 and si-FOXO1 NC (si-NC) were obtained from RIBO Bio (Guangzhou, China). CCRF-CEM and NALM-6 cells grown to 80% confluence were transfected or co-transfected with these above agents using Lipofectamine 3000 (Invitrogen). The CCRF-CEM and NALM-6 cells were randomly divided into NC-mimic group (transfected with NC-mimic), miR-223 mimic group (transfected with miR-223 mimic), NC-inhibitor group (transfected with NC-inhibitor) and miR-223 inhibitor group (transfected with miR-223 inhibitor). In addition, the NALM-6 cells were randomly divided into si-NC group (transfected with si-NC), si-FOXO1-1 group (transfected with si-FOXO1-1), si-FOXO1-2 group (transfected with si-FOXO1-2), si-NC + NC-inhibitor group (co-transfected with si-NC and NC-inhibitor), si-FOXO1 + NC-inhibitor group (co-transfected with si-FOXO1 and NC-inhibitor) and si-FOXO1 + miR-223 inhibitor group (co-transfected with si-FOXO1 and miR-223 inhibitor). Cells without transfection were considered as the BLANK (BLANK group). All cells were cultured in 37°C incubator for 48 h.

RETRACTED

### Dual luciferase reporter gene assay

The potential binding site of miR-223 on FOXO1 was predicted by TargetScan. FOXO1 with WT or MUT miR-223-binding sites were generated and cloned into pmirGLO vector (Promega, Madison, WI, U.S.A.) (FOXO1-WT and FOXO1-MUT). FOXO1-WT/FOXO1-MUT were then co-transfected with miR-223 mimic/NC-mimic into CCRF-CEM and NALM-6 cells with Lipofectamine 3000 (Invitrogen) for 48 h. The luciferase activity was detected by dual-luciferase reporter gene assay system (Promega).

### RNA pull-down assay

Biotinylated FOXO1 (Bio-FOXO1-Wt), FOXO1-Mut (Bio-FOXO1-Mut) and NC (Bio-NC) were purchased from GenePharma and were transfected into CCRF-CEM and NALM-6 cells. After 48 h of transfection, the cells were lysed and then incubated with Streptavidin agarose beads (Invitrogen) at 37°C for 1 h. In the end, qRT-PCR assay was employed to assess the enrichment of miR-223.

### Western blot

CCRF-CEM and NALM-6 cells were lysed by ice-cold lysis buffer to obtain total protein. Protein concentration was detected by Bicinchoninic Acid Kit (CST, Danvers, MA, U.S.A.). Protein samples were separated in SDS-PAGE, and transferred onto nitrocellulose membrane. Then membranes were incubated with primary antibody overnight at 4°C. The antibodies were shown as follows: anti-FOXO1 (1:1000, ab52857, Abcam, Cambridge, MA, U.S.A.). The membranes were subsequently incubated with secondary antibody, horseradish peroxidase (HRP)-labeled goat anti-rabbit IgG (1:2000, 12-348MSDS, Sigma) for 1 h at 25°C. The protein bands were visualized by enhanced chemiluminescence (ECL) exposure solution, and quantified by Quantity One 1-D software (Bio-Rad, Hercules, CA, U.S.A.). α-Tublin (1:1000, MABT205, Sigma) was introduced as the internal reference.

### MTT assay

The proliferation of CCRF-CEM and NALM-6 cells were tested by MTT Kit (Sigma, St. Louis, MO, U.S.A.). In brief, the transfected cells (2 × 10^4^ cells/well) were planted into 96-well plates. MTT (20 μl) was added into each well at 0, 24, 48, 72 and 96 h. Subsequently, the cells were then cultured at 25°C for 1 h. The absorbance was measured at 450 nm by a microplate reader (Bio-Rad).

### Colony formation assay

The transfected CCRF-CEM and NALM-6 cells were respectively seeded into six-well plates (300 cells/well) and cultivated for 14 d. After fixed in 4% cold formaldehyde for 30 min, the colonies were stained with 0.1% Crystal Violet (Sigma) for 20 min. The colonies were photographed and counted under an optical microscope (Olympus, Tokyo, Japan).

RETRACTED

### Flow cytometer

The transfected CCRF-CEM and NALM-6 cells were collected and resuspended in binding buffer. Then, the transfected cells were stained by using Annexin V-FITC and propidium iodide (Invitrogen) for 15 min in a dark room. Subsequently, the apoptotic cells were observed by MUSE™ flow cytometer (Beckman, Miami, FL, U.S.A.).

### Transwell assay

The transwell assay was performed to determine the cell invasion and migration by using transwell chambers (8 nm pore size) (Corning Inc., Corning, NY, U.S.A.). The transfected cells at a density 1 × 10^5^ cells/well were inoculated to the upper chamber covered with Matrigel (BD Biosciences, San Jose, CA, U.S.A.). Then RPMI–1640 medium with 10% FBS was added into the lower chamber. After incubation for 24 h at 37°C, the CCRF-CEM and NALM-6 cells were removed from the upper chambers with a cotton swab, and cells in lower chambers were fixed with 4% paraformaldehyde and stained with 0.5% Crystal Violet dye (Sigma, U.S.A.) for 30 min at room temperature. After washing three times, the number of invasion and migration cells was calculated under an optical microscope (200×).

### Statistical analysis

All statistical analyses were performed using SPSS 22.0 Statistical software (Chicago, IL, U.S.A.) and GraphPad Prism 7.0 software (GraphPad, San Diego, CA, U.S.A.). The results were presented as the mean ± SD. All experiments were carried out at least three times. The differences between two groups were assessed using the Student’s *t-*test. The differences among multiple groups were analyzed by one-way ANOVA followed by the Tukey’s post hoc test. The differences on cell proliferation at different time points were analyzed by repeated measurement ANOVA. *P*<0.05 was considered to be statistically significant.

## Results

### The expression of miR-223 was down-regulated in ALL children

The mRNA expression of miR-223 in 59 ALL children and 30 control children was detected by qRT-PCR. The miR-223 expression was markedly reduced in the ALL group compared with the Control group (*P*<0.001). The expression of miR-223 in the IR-ALL group was significantly lower than that in the SR-ALL group, and the expression of miR-223 in the HR-ALL group was dramatically lower than that in the IR-ALL group (all *P*<0.05). The results indicated that the expression of miR-223 was down-regulated in ALL children, especially in the HR-ALL group (children with high risk) (Figure 1A). The receiver operating characteristic (ROC) curve was plotted to evaluate the diagnostic value of miR-223 in ALL. We obtained a highly significant area under curve (AUC) which gave a good separation between Control and ALL (sensitivity is 93.22% and specificity is 93.33%, *P*<0.0001) (Figure 1B and Table 2). ROC curve analysis also confirmed that miR-223 has diagnostic value to distinguish Control and SR-ALL (sensitivity is 94.12% and the specificity is 76.67%, *P*<0.0001) (Figure 1C and Table 2). In addition, miR-223 has limited diagnostic value to distinguish SR-ALL and IR-ALL because of the low sensitivity (36.00%) (Figure 1D and Table 2), and miR-223 has limited diagnostic value to distinguish IR-ALL and HR-ALL because of the low specificity (48.00%) (Figure 1E and Table 2), miR-223 has limited diagnostic value to distinguish SR-ALL and HR-ALL because of the low specificity (64.71%) (Figure 1F and Table 2). As shown in Table 3, miR-223 expression had no connection with gender, age and immunophenotype in ALL children (*P*>0.05). Moreover, the miR-223 expression was related to WBC, PLT, RBC and risk stratification in ALL children (*P*<0.001).

RETRACTED

**Figure 1:** The expression of miR-223 was down-regulated in acute lymphoblastic leukemia (ALL) children (**A**) qRT-PCR was conducted to detect the miR-223 expression. ***P<0.001 vs*.* Control; ^#^*P*<0.05, ^##^*P*<0.01 vs*.* SR-ALL; ^&^*P*<0.05 vs*.* IR-ALL. (**B–F**) The receiver operating characteristic (ROC) curve was plotted to evaluate the diagnostic value of miR-223 in ALL children.

**Table 2:** Results of the ROC analysis for miR-223

Group	Cut off	Sensitivity (%)	Specificity (%)	AUC (Area ± Std. Error)	95% CI	*P* value
Control vs.ALL	0.705	93.22	93.33	0.978 ± 0.013	0.953–0.999	<0.0001
Control vs.SR-ALL	0.875	94.12	76.67	0.952 ± 0.028	0.898–0.999	<0.0001
SR-ALL vs.IR-ALL	0.395	36.00	94.12	0.707 ± 0.080	0.550–0.865	0.0241
IR-ALL vs.HR-ALL	0.465	82.35	48.00	0.681 ± 0.081	0.522–0.841	0.0485
SR-ALL vs.HR-ALL	0.510	88.24	64.71	0.870 ± 0.059	0.755–0.985	0.0002

**Table 3:** Correlation between miR-223 expression and clinical characteristics in ALL children

	*N*	miR-223 expression	*P* value
Gender			0.8531
Male	29	0.457 ± 0.192	
Female	30	0.448 ± 0.175	
Age (Year)			0.7097
<10	36	0.459 ± 0.196	
10∼18	23	0.441 ± 0.160	
WBC(×10^9^/l)			<0.0001
<50	20	0.610 ± 0.159	
≥50	39	0.371 ± 0.135	
PLT(×10^9^/l)			<0.0001
<100	31	0.320 ± 0.117	
≥100	28	0.599 ± 0.115	
RBC(×10^12^/l)			0.0005***
<4	27	0.366 ± 0.180	
≥4	32	0.525 ± 0.151	
Immunophenotype			
B-ALL	27	0.466 ± 0.194	0.5943
T-ALL	32	0.440 ± 0.173	
Risk stratification			
SR-ALL	17	0.583 ± 0.158	0.0002***
IR-ALL	25	0.440 ± 0.171	
HR-ALL	17	0.338 ± 0.137	

***P<0.001. Abbreviations: PLT, blood platelet; RBC, red blood cell; WBC, white blood cell.

### MiR-223 inhibited the cell proliferation, colony formation ability and promoted cell apoptosis in ALL

Firstly, miR-223 was overexpressed by the transfection of miR-223 mimic, and blocked by the transfection of miR-223 inhibitor into CCRF-CEM and NALM-6 cells. (*P*<0.01) (Figure 2A). MTT assay showed that the OD_450_ value of CCRF-CEM cells in the miR-223 mimic group was markedly decreased compared with the NC-mimic group at 48 h (*P*<0.05), 72 h (*P*<0.01) and 96 h post-culturing (*P*<0.01). The OD_450_ value of NALM-6 cells in the miR-223 inhibitor group was higher than that in the NC-inhibitor group at 48 h (*P*<0.05), 72 h (*P*<0.01) and 96 h post-culturing (*P*<0.01) (Figure 2B). Colony formation assay confirmed that miR-223 mimic markedly decreased the number of cell colonies of CCRF-CEM cells, and miR-223 inhibitor markedly increased the number of cell colonies of NALM-6 cells (*P*<0.01) (Figure 2C). In addition, flow cytometry displayed that the apoptosis of CCRF-CEM cells in the miR-223 mimic group was significantly increased compared with the NC-mimic group, the apoptosis of NALM-6 cells in the miR-223 inhibitor group was dramatically decreased compared with the NC-mimic group (*P*<0.01) (Figure 2D).

RETRACTED

**Figure 2:** miR-223 inhibited the cell proliferation, colony formation ability and promoted cell apoptosis in ALL (**A**) The mRNA expression of miR-223 in CCRF-CEM and NALM-6 cells was detected by qRT-PCR. (**B**) The OD_450_ value of CCRF-CEM and NALM-6 cells was determined by MTT assay. (**C**) The number of CCRF-CEM and NALM-6 cell colonies was confirmed by colony formation assay. (**D**) The apoptosis of CCRF-CEM and NALM-6 cells was detected by flow cytometry. **P<0.01 vs. NC-mimic; ^##^*P*<0.01 vs*.* NC-inhibitor.

### MiR-223 inhibited the cell invasion and migration in ALL

Transwell assay was used to detect the migration and invasion of ALL cells. As shown in Figure 3A, the number of migration cells was dramatically decreased by the transfection of miR-223 mimic in CCRF-CEM cells (*P*<0.01), and was dramatically increased by the transfection of miR-223 inhibitor in NALM-6 cells (*P*<0.01). The number of invasion cells was dramatically reduced by the transfection of miR-223 mimic in CCRF-CEM cells (*P*<0.01), and was dramatically elevated by the transfection of miR-223 inhibitor in NALM-6 cells (*P*<0.01) (Figure 3B).

**Figure 3:** miR-223 inhibited the cell invasion and migration in ALL (**A** and **B**) The number of invasion and migration cells in CCRF-CEM and NALM-6 cells was measured by transwell assay; magnification, ×200) **P<0.01 vs. NC-mimic group; *^##^P*<0.01 *vs.* NC-inhibitor group.

### MiR-223 inhibited the protein expression of FOXO1 in ALL cells

As shown in Figure 4A, TargetScan predicted a binding site for miR-233-3p in the FOXO1 3′ UTR. The expression of FOXO1 in 59 cases of ALL children and 30 control children was detected by qRT-PCR. The expression of FOXO1 was dramatically up-regulated in the ALL group compared with the Control group (*P*<0.001). The expression of FOXO1 in the IR-ALL group was dramatically higher than that in the SR-ALL group, and the expression of FOXO1 in the HR-ALL group was dramatically higher than that in the IR-ALL group (all *P*<0.05). The results indicated that the FOXO1 expression was increased in ALL children, especially in the HR-ALL group (Figure 4B). We also found that miR-223 expression was negatively correlated with the expression of FOXO1 in ALL (*r* = −0.4311, *P*=0.0007) (Figure 4C). Next, dual-luciferase reporter assay showed that the relative luciferase activity was markedly decreased in CCRF-CEM and NALM-6 cells co-transfected with miR-223 mimic and FOXO1-Wt compared with cells co-transfected with NC-mimic and FOXO1-Wt (*P*<0.01) (Figure 4D). RNA-pull down assay showed that the expression of miR-223 in CCRF-CEM and NALM-6 cells in the FOXO1-Wt group was markedly increased compared with the Bio-NC group (*P*<0.01) (Figure 4E). Furthermore, Western blot showed that overexpression of miR-223 decreased the FOXO1 protein expression in CCRF-CEM cells (*P*<0.01) (Figure 4F), and transfection of miR-223 inhibitor increased the FOXO1 protein expression in NALM-6 cells (*P*<0.01) (Figure 4G).

RETRACTED

**Figure 4:** miR-223 inhibited the protein expression of FOXO1 in ALL cells (**A**) The binding target of miR-223 on FOXO1 was predicted by TargetScan software. (**B**) The expression of FOXO1 in ALL children and control children was detected by qRT-PCR. ***P<0.001 vs. Control; ^#^*P*<0.05, ^##^*P*<0.01 vs. SR-ALL; ^&^*P*<0.05 vs. IR-ALL. (**C**) The expression of miR-223 was negatively correlated with FOXO1 in ALL. (**D**) Relative luciferase activity in CCRF-CEM and NALM6 cells was measured by dual-luciferase reporter assay; **P<0.01 vs. NC-mimic group. (**E**) The interaction of FOXO1 and miR-223 in CCRF-CEM and NALM-6 cells was detected by RNA pull-down assay; **P<0.01 vs. Bio-NC. (**F** and **G**) The protein expression of FOXO1 in CCRF-CEM and NALM-6 cells was detected by Western blot; **P<0.01 vs. NC-mimic.

### FOXO1 reversed the inhibiting effect of miR-223 on the tumorigenesis of ALL

To further explore whether FOXO1 is involved in the role of miR-223 in ALL cells, si-FOXO1-1 and si-FOXO1-2 were transferred into NALM-6 cells. The protein expression of FOXO1 was dramatically down-regulated in NALM-6 cells after transfected with si-FOXO1-1 and si-FOXO1-2 (*P*<0.01) (Figure 5A). Then si-FOXO1-1 was used for subsequent assays. To explore whether miR-223 exerted its function in ALL through regulating FOXO1, NALM-6 cells were co-transfected with si-FOXO1 and miR-223 inhibitor. Compared with the si-NC + NC inhibitor group, the OD_450_ value of NALM-6 cells was markedly reduced in the si-FOXO1 + NC inhibitor group at 72 and 96 h post-culturing (*P*<0.01). The transfection of si-FOXO1 markedly reversed the promoting effect of miR-223 inhibitor on the OD_450_ value (*P*<0.01) (Figure 5B). Compared with the si-NC + NC inhibitor group, the number of cell colonies, numbers of migrant and invasive cells of NALM-6 cells were markedly increased in the si-FOXO1 + NC inhibitor group (*P*<0.01). Transfection of si-FOXO1 markedly reversed the promoting effect of miR-223 inhibitor on the above indexes in NALM-6 cells (*P*<0.001) (Figure 5C,E,F). In addition, the apoptosis of NALM-6 cells was contrary with OD_450_ value (*P*<0.01) (Figure 5D).

RETRACTED

**Figure 5:** FOXO1 reversed the effects of miR-223 in ALL cells (**A**) The protein expression of FOXO1in NALM-6 cells was detected by Western blot; **P<0.01 vs. si-NC. (**B**) The OD_450_ value of NALM-6 cells was determined by MTT assay. (**C**) The number of NALM-6 cell colonies was confirmed by colony formation assay. (**D**) The apoptosis of NALM-6 cell colonies was measured by flow cytometry. (**E** and **F**) The numbers of migration and invasion cells of NALM-6 cells were measured by transwell assay (magnification, ×200); **P<0.01 vs. si-NC + NC-inhibitor; ^##^*P* < 0.01vs. si-FOXO1 + NC-223 inhibitor.

## Discussion

ALL is a hematological malignant tumor characterized by dysplastic lymphoid cells and abnormal differentiation, resulting in the formation of a large number of immature leukocytes [18]. Abnormal expression of miRNAs is related to the tumorigenesis of ALL. The expression of some miRNAs such as miR-196b [19], miR-509 [20] and miR-101 [21] was decreased in ALL patients. Similar to the previous studies, miR-223 expression was markedly reduced in ALL children in the present study. We suspect that miR-223 plays a critical part in inhibiting the tumorigenesis of ALL. Some miRNAs are important diagnostic markers for ALL [22,23]. For instance, higher miR-708-5p expression was related to WBC in ALL patients [24]. Up-regulation of miR-29 markedly increased the percent of PLT in patients with T-cell ALL [25]. Overexpression of miR-200a was related to the risk stratification in children with B-cell ALL [26]. In the present study, overexpression of miR-223 was related to the numbers of WBC, PLT, RBC and risk stratification in ALL children. The function of miR-223 was similar to the above miRNAs. MiR-223 may be a valuable diagnostic marker for ALL. In addition, ROC curve analysis reconfirmed that miR-223 has diagnostic value to distinguish Control and ALL or SR-ALL. However, miR-223 was limited in distinguishing ALL with different risk (SR, IR and HR). MiR-223 may be used as an auxiliary diagnostic marker for ALL. Because the Control group did not include malignant hematologic diseases other than ALL, these diseases may limit the diagnostic value of miR-223 in clinical practice. Further researches on the diagnostic value of miR-223 in ALL are still needed.

RETRACTED

The down-regulation of miR-223 has been discovered in different cancers, such as esophageal carcinoma [27], hepatocellular carcinoma [28], and osteosarcoma [29]. These researches have proved that miR-223 has anticancer effect. More and more researches have displayed that miR-223 can not only attenuate cell growth and metastasis, but also promote cell apoptosis in leukemia. Li et al. have proved that miR-223 prevents the malignant biological behavior of ALL cells via regulating MAPK signal pathway and Lmo2 [30]. Jia et al. have suggested that miR-223 reduces the proliferation of leukemia cells through targeting IGF-1R [31]. Xiao et al. have found that miR-223 accelerates the apoptosis of acute myeloid leukemia (AML) cells by targeting FBXW7 [32]. Here, up-regulation of miR-223 inhibited the proliferation, migration and invasion of ALL cells, and promoted the apoptosis. Our research suggests that miR-223 protects children against ALL through attenuating the proliferation, migration, and invasion of ALL cells and promoting apoptosis. Based on these studies, up-regulation of miR-223 may be a novel target for the treatment of ALL.

The expression of FOXO family members is highly expressed in leukemia, such as FOXO3A in AML [33] and FOXO1 in most of the B-cell precursor (BCP)-ALL cell lines [34]. Similar to the previous studies, the expression of FOXO1 was increased in ALL children in the present study. FOXO family members are important mediators in leukemia development. For instance, FOXO family members contribute to leukemogenesis through maintaining leukemia stem cells and stimulating drug resistance genes [35]. FOXO proteins promote tumor cell growth and maintenance in AML and chronic myeloid leukemia [36]. FOXO1 serves as a tumor promoter in human CD34^+^ cells and accelerates preleukemia transition [37]. FOXO1 usually exerts its function in regulating the tumorigenesis as a downstream target of miRNAs [38,39]. In the present study, FOXO1 was a target of miR-223, and the expression of FOXO1 negatively related to miR-223 in ALL. We suspect that miR-223 participates in the development of ALL via targeting FOXO1. In addition, our results displayed that FOXO1 markedly reversed the effects of miR-223 on inhibiting cell proliferation, colony formation ability, migration and invasion, and promoting apoptosis in ALL children. To sum up, miR-223 may protect children against the development of ALL through inhibiting the expression of FOXO1.

RETRACTED

In conclusion, our results confirmed that miR-223 expression was down-regulated in ALL. Moreover, miR-223 could inhibit cell proliferation and promote apoptosis in ALL children via regulating FOXO1. Our research indicated that miR-223 might act as a potential therapeutic target for ALL. However, the detailed action mechanism of miR-223 on ALL remains limited, and further research is still needed.

## Data Availability

The data contained in this study can be obtained from the corresponding author with the permission of the corresponding author’s institution

## Abbreviations

ALL: acute lymphoblastic leukemia
AML: acute myeloid leukemia
BCP: B-cell precursor
CLL: chronic lymphocytic leukemia
ECL: enhanced chemiluminescence
FBS: fetal bovine serum
FOXO: Forkhead box class O
HR: high risk
IR: intermediate risk
miRNA: microRNA
NC: negative control
SR: standard risk
